# Research on the Impact of Entrepreneurship Education on Employee Creativity from the Perspective of Career Environment Based on an Intermediary Model

**DOI:** 10.1155/2022/1677620

**Published:** 2022-08-08

**Authors:** Heli Wang, Runkai Jiao, Feifei Li

**Affiliations:** School of Psychology, Northeast Normal University, Changchun 130024, China

## Abstract

Based on the human capital theory and creativity component theory, this study empirically examines the direct effect of entrepreneurship education on employees' environment protection creativity in the workplace and the dual mediating effect of boundary-free mental model and organizational mobility preference based on 266 valid sample data. The results show that entrepreneurship and environmental protection education received in colleges and universities can significantly promote the improvement of employees' environment protection creativity. Borderless mental model and organizational mobility preference play an intermediary role between them. The impact of entrepreneurship education on creativity is expanded from college students to employees through the bridge of borderless career attitude, which effectively verifies the lag effect of entrepreneurship education in colleges and universities and the dual intermediary effect of borderless mental model and organizational mobility preference. It further expands the research on the impact of entrepreneurship education in colleges and universities and has certain theoretical value.

## 1. Introduction

In 2017, China's concept of “mass entrepreneurship and innovation” was written into the UN resolution, which shows that innovation and entrepreneurship have become an international consensus in driving economic growth and social progress. In order to meet the needs of economic development in the new era, as one of the important ways to cultivate creative talents, entrepreneurship education has risen to a strategic height at the national level, which requires universities to carry out for all students and run through the whole process of talent training systematically. According to the 2017 survey, the rate of college students starting businesses in China has reached 3 percent, much higher than the average of 1.6 percent in developed countries. Despite the remarkable results of entrepreneurship education in colleges and universities, the vast majority of students who have received good entrepreneurship education at school always prefer to work in enterprise rather than to start a business after graduation. So, if most students do not start businesses, why teach them about entrepreneurship? Is this a waste of educational resources?

In order to answer the above questions, we must clearly recognize that entrepreneurship education is not only to improve the entrepreneurial rate of college students but also to cultivate the entrepreneurial spirit of students. The spirit of entrepreneurship is mainly manifested in innovation, risk tolerance, unity and cooperation, perseverance, and other fine qualities. The Basic Requirements for Entrepreneurship Education and Teaching in Ordinary Undergraduate Schools (Trial) formulated by the Ministry of Education in 2012 clearly points out that students' innovative consciousness and thinking should be cultivated through entrepreneurship education. Therefore, entrepreneurship education in colleges and universities is crucial for students to carry out entrepreneurship and innovation in the future. However, existing studies mainly focus on the impact of entrepreneurship education on entrepreneurship, including entrepreneurial self-efficacy, entrepreneurial ability, entrepreneurial willingness, and entrepreneurial behavior, but ignore its impact on innovation. As a large number of college students with systematic entrepreneurship education enter the workplace and become the source of enterprise innovation, how to give full play to the lagged effect of college entrepreneurship education on enterprise creative talent training and open the “black box” of the relationship between college entrepreneurship education and enterprise employees' creativity in the workplace has become an urgent issue to be explored in the current college entrepreneurship education.

Creativity is the basis of individual innovation [1]. Although some scholars have explored the impact of entrepreneurship education in colleges and universities on creativity, most of them focus on college students, who have not yet entered the workplace, and their creativity is greatly different from that of workplace in application context and expression form. Workplace creativity refers to innovative and practical ideas put forward by employees for work and organization [2]. The creativity component theory of Amabile [2] points out that whether an individual has domain-related skills, creativity and intrinsic motivation will affect his or her creative performance. According to the human capital theory, entrepreneurship education, which mainly focuses on cultivating the basic ability of innovation and entrepreneurship and mainly aims at meeting the quality requirements of innovative talents, creates conditions for employees to improve their skills and creativity in the work field through resource and skill accumulation.

In addition, the Basic Requirements for Entrepreneurship Education in Ordinary Undergraduate Schools (Trial) clearly points out that students should be aware of the positive role of entrepreneurship education in their own career development. Entrepreneurship education in colleges and universities does not expect all educated students to start their own businesses. It only provides a choice for college students in career development planning, and its essence is to broaden the realization of human subject value. In the era of borderless career, there are more and more work intersections among employees of different organizations or departments [3]. Job-related creativity no longer follows the cultivation mode of closed door but requires employees to communicate across organizational boundaries and constantly update their work fields and creativity-related skills. Therefore, the attitude of employees towards borderless career is very important, and this occupation tendency is not only the value orientation advocated by entrepreneurship education in colleges and universities but also the innovative motivation internalized by entrepreneurship. Therefore, this paper argues that borderless career attitude plays an importantly intermediary role in the delayed impact of entrepreneurship education on employees' workplace creativity. Borderless career attitude includes two dimensions: borderless mental model and organizational mobility preference [3]. Although both mental model and organizational mobility preference represent the psychological tendency of individuals to work across borders, there are essential differences. Although employees with borderless mental model are keen on cross-border cooperation with others, they still stay in their current organization, while employees with preference for organizational mobility will serve other organizations outside their current organization.

## 2. Theoretical Basis and Research Hypothesis

### 2.1. College Entrepreneurship Education and Employee Creativity

Entrepreneurship education aims to cultivate students' entrepreneurial spirit, consciousness, and ability. Compared with professional education, entrepreneurship education is not limited to a specific education stage but to an educational orientation that runs through life and is oriented to the development of all mankind. In the teaching practice of colleges and universities, innovation and entrepreneurship education are often difficult to separate, because the entrepreneurial process is a series of creative activities. Therefore, entrepreneurship education is bound to include skills related to creativity, and good entrepreneurship education received by employees in college contributes to the improvement of their workplace creativity.

From the perspective of cognition, according to the creativity component theory of Amabile [2], domain-related skills, innovation skills, and internal motivation are the raw materials for the formation of employees' creativity. By integrating the concept of innovation and entrepreneurship education into professional education, entrepreneurship education helps students build a cognitive system and make comprehensive use of professional knowledge and innovative skills, so as to improve their problem-solving ability after work. In terms of internal motivation, entrepreneurship education stimulates employees' autonomy to explore, analyze, and solve problems by cultivating employees' entrepreneurial thinking. When Yang Tao analyzed the work motivation of employees of different generations, he found that compared with other employees, the new generation of employees explored more independently, learned new things more frequently and in greater depth, and had stronger intrinsic motivation. According to the motivational information processing theory, employees with high level of intrinsic motivation are more willing to challenge high goals, more motivated to complete creative and systematic information processing work [4], and more willing to try and learn new ways to solve problems [5]. From the perspective of social learning, entrepreneurship education helps the new generation of employees accumulate innovative knowledge and resources, so as to improve their innovative self-efficacy [6]. Innovative self-efficacy helps employees resolve work pressure by giving them the belief to solve problems at work, improve their sense of psychological security, and maintain a positive working state, so as to help stimulate their creative cognition and creative behavior. Therefore, this paper proposes the following hypothesis:

  H1: Entrepreneurship education received in colleges and universities is positively correlated with employee creativity.

### 2.2. The Mediating Role of Borderless Mental Models

Boundary-free career attitude, first proposed by Arthur [7, 8], refers to an individual's attitude when choosing and managing career opportunities beyond a single employer or work boundary. It focuses on individual's flexibility, adaptability, and self-assessment in career development behavior, so as to achieve career success [9]. Borderless mental model, as one of the manifestations of borderless occupational attitude, reflects the individual's psychological preference and ability to spontaneously pursue boundary-spanning work relationships. Employees with boundless mental models tend to pursue working relationships across departments and organizational boundaries and are keen on establishing and maintaining positive relationships outside departments and organizations [3].

Studies show that education can influence the choice of individual career mode, and individuals with higher education level prefer the borderless career mode [10]. The ultimate goal of entrepreneurship education is to cultivate individual entrepreneurship, which plays an important role in shaping the borderless mental model of the new generation of employees. The so-called entrepreneurial spirit refers to the thinking mode of transforming innovative ideas into innovative practice planning under the guidance of innovative spirit. The new generation of employees with entrepreneurial spirit has both openness and rational cognition of opportunities and is good at reshaping resources and systems [11]. In addition, entrepreneurship education focuses on career guidance, which helps students to consider their future choices more actively after they start to work, develop their vocational adaptability, and accumulate social capital [3], so as to strengthen their sense of responsibility and cooperation to share experience and knowledge across borders. Therefore, the new generation of employees with entrepreneurial education experience tends to be more sensitive and open to working relationships across organizational or departmental boundaries.

Borderless mental model, as a professional value, is closely related to the creativity of the new generation of employees. Directly, the new generation of employees with borderless mental model is keen on creating and maintaining positive relationships outside the boundaries of the organization [3], so they are more likely to obtain professional support [12, 13] to provide conditions for their creativity. Indirectly, on the one hand, employees with borderless mental model have higher career satisfaction and easier access to emotional support, so as to achieve a positive emotional state [13]. Studies have shown that people have more creative thinking in a positive emotional state [14]. On the other hand, individuals with borderless mental models have a higher tolerance for uncertainty and ambiguity and are more willing to try highly innovative solutions at work [15]. In addition, Andresen and Margenfeld [16] believed that employees with borderless mental model are more likely to experience job transfer across functional departments. By establishing new working relationships, expanding social networks and cross-departmental mobility, the new generation of employees can accumulate experience in different fields and work roles [17], improve their skills and creativity in their work fields, and further stimulate their internal motivation for innovation. Therefore, this paper proposes the following hypotheses:

  H2: Entrepreneurship education received in colleges and universities is positively correlated with the borderless mental model of the new generation of employees.
  H3: The borderless mental model of the new generation of employees is positively correlated with creativity.
  H4: The borderless mental model of the new generation of employees plays an intermediary role in the relationship between entrepreneurship education and creativity.

### 2.3. The Mediating Role of Organizational Mobility Preference

Organizational mobility preference is another manifestation of borderless professional attitude, which refers to the psychological tendency of individuals to cross-border “real” and “physical” work flow [3]. The most essential difference between organizational mobility preference and borderless mental model is that although individuals with borderless mind are keen to cross-border cooperation with people, they will still stay in the current organization, and individuals with organizational mobility preference will serve other organizations in addition to the current organization. Employees with strong organizational mobility preference are more adaptable and even appreciate jobs that require competition among multiple employers [3], thus affecting employees' preference for crossing specific occupational boundaries. Previous studies have shown that education will affect individual employees' borderless professional attitudes, and employees with higher education usually benefit more from borderless professional attitudes [18]. Entrepreneurship education affects employees' willingness to flow among organizations by cultivating their employment concept and entrepreneurial spirit. First of all, one of the goals of entrepreneurship education is to change students' employment concept and career choice concept. Compared with professional education, entrepreneurship education helps to cultivate students' ability of rational career choice so that they can actively consider their future career choice and get rid of the career vacuum. Therefore, employees with entrepreneurship education have very clear career goals and plans before entering the organization and are not likely to change jobs frequently after entering the organization. Secondly, entrepreneurship education in colleges and universities cultivates the entrepreneurial spirit of students, who tend to have stronger promotion motivation rather than prevention motivation in career development and pay more attention to career development rather than occupational safety. According to the theory of adjusting focus, controlling focus motivation can shape employees' career attitude [19]. Employees with strong promotion motivation have higher career concentration and adaptability to occupational environment, and their organizational mobility preference tends to be lower.

Existing studies have shown that organizational mobility preference inhibits individual creativity. From an objective point of view, employees with high organizational mobility preference prefer to work for different organizations than those who only work for their current employer. On the one hand, these employees are less willing to make internal investment in their existing careers [20]; On the other hand, employers tend to reduce career support and resource investment for employees with strong organizational mobility preferences [21]. Therefore, the lack of self-career investment and organizational career support will have a negative impact on employee creativity. From the subjective perspective, employees with strong organizational mobility preference usually have lower career satisfaction [22, 23]. Low level of career satisfaction is more likely to stimulate employees' negative emotions. According to the theory of emotional expansion-construction, negative emotions limit the activity space and cognitive scope of individual thinking, thus inhibiting the improvement of employees' creativity [14]. Therefore, this paper proposes the following hypotheses:

  H5: Entrepreneurship education received in colleges and universities is negatively correlated with employees' preference for organizational mobility.
  H6: Employees' organizational mobility preference is negatively correlated with creativity.
  H7: Employees' organizational mobility preference plays an intermediary role in the relationship between entrepreneurship education and creativity.

To sum up, the research model constructed in this paper is shown in Figure 1.

## 3. Research Design

### 3.1. Research Samples

Since the 17th National Congress of the Communist Party of China in 2007 proposed the idea of “entrepreneurship to promote employment,” colleges and universities across the country have actively promoted entrepreneurship education. Taking Jiangsu Province as an example, by the end of 2008, 85% of colleges and universities had set up entrepreneurship education courses. In 2012, the Ministry of Education formulated the Basic Requirements for Entrepreneurship Education and Teaching in Ordinary Undergraduate Schools (Trial), requiring colleges and universities to carefully organize and carry out entrepreneurship education and teaching activities. The knowledge workers of the new generation after 1990 not only have generally received entrepreneurship education but also have different degrees of completeness in receiving entrepreneurship education. This group as the research object can obtain great variation in the measurement of entrepreneurial education perception, which is conducive to better solve the research problem. In January 2019, this study recruited post-90s knowledge workers with higher education to participate in the questionnaire survey. In order to improve the quality and recovery rate of the questionnaire, participants who effectively completed the questionnaire were promised a certain amount of cash reward. At the same time, in order to effectively avoid the problem of homologous variance, this study collects data at three time points. A total of 350 questionnaires were distributed for the first time, which mainly collected the respondents' personal information and their subjective perception data of entrepreneurship education received during the university, and a total of 336 questionnaires were recovered. One month later, 301 questionnaires were collected from the participants who answered the questionnaire for the first time. The data were mainly collected on employees' borderless career attitude (borderless mental model and organizational mobility preference). One month later, a questionnaire was sent to the participants who answered the questionnaire for the second time, mainly collecting employee creativity data and relevant information of their enterprises. A total of 283 questionnaires were recovered. After further eliminating the invalid questionnaires, 266 valid questionnaires were finally obtained, with an effective recovery rate of 76.00 (266/350), as shown in Table 1.

### 3.2. Measuring Tools

The main variables of this study were measured by the Western maturity scale, which strictly followed the translation and back-translation procedures. Firstly, two scholars in the field of entrepreneurship and management jointly translated the English items into Chinese and then back-translated the Chinese items into English until the back-translated items were clear and consistent with the original English. The measurement was measured by the 5-point Likert scoring method.

#### 3.2.1. Entrepreneurship Education in Colleges and Universities (Cronbach's *α* = 0.840)

The 4-item scale developed by Walter and Block [24] was used to measure the subjective experience of entrepreneurship education received by individuals in colleges. The reliability and validity of the scale have been verified in the Chinese context.

#### 3.2.2. Borderless Career Attitude

Borderless career attitude was measured using a 13-item two-dimensional scale developed by Briscoe et al. [3], which has been widely used in the Chinese context. Among them, the first 8 items measured the dimensionality of borderless mental model (Cronbach's *α* = 0.863), and the last five items measured the dimensionality of organizational mobility preference (Cronbach's *α* = 0.839).

#### 3.2.3. Creativity (Cronbach's *α* = 0.863)

The 6-item scale developed by Grant [25] was used for measurement, which has been widely used by scholars in the Chinese context and has good reliability and validity.

#### 3.2.4. Control Variables

Existing studies have shown that factors such as gender, age, education level, working years, position, enterprise size, and nature of employees have an impact on the dependent variable creativity. Therefore, it is treated as a control variable in this study.

## 4. Hypothesis Testing and Result Analysis

### 4.1. Common Method Deviation Test

Although the data in this study were collected at different time points, they were all filled in by the same object. Therefore, it is necessary to adopt Harman's single-factor test to test common method deviation before hypothesis testing. The unrotated principal component analysis precipitated four factors with eigenvalues > 1, and the first factor explained the variance of 33.042, which was less than the critical point of 50. It can be seen that there is no serious common method bias in the sample data.

### 4.2. Correlation Analysis

The results of correlation analysis of main variables in this study are shown in Table 2. Entrepreneurship education received by employees in colleges and universities is significantly positively correlated with workplace creativity (*r* = 0.377, *P* < 0.01). Entrepreneurship education received by employees in colleges and universities was significantly positively correlated with borderless mental model (*r* = 0.442, *P* < 0.01) but negatively correlated with organizational mobility preference (*r* = −0.365, *P* < 0.01). Borderless mental model was significantly positively correlated with employees' workplace creativity (*r* = 0.563, *P* < 0.01), while organizational mobility preference was significantly negatively correlated with employees' workplace creativity (*r* = −0.316, *P* < 0.001). It can be seen that the research hypothesis has been preliminarily supported and is suitable for further hypothesis testing.

### 4.3. Confirmatory Factor Analysis

In this study, confirmatory factor analysis (CFA) was used to investigate the differentiability among major variables. Considering that there are many measurement items for some variables and the effective sample size is small, in order to improve the overall model fitting degree, the borderless mental model and creativity measurement items are packaged separately according to the suggestion of Little et al. [26] before the implementation of CFA. After packaging, the results of CFA are shown in Table 3, and the fitting indexes of the 4-factor benchmark model (*χ*^2^ = 151.756, Df = 84, *χ*^2^/Df = 1.807, GFI = 0.930, TLI = 0957, CFI = 0.966, RMSEA = 0.055) were significantly better than those of the competition model, which fully indicated that there was a high degree of differentiation among the four variables.

### 4.4. Hypothesis Testing

#### 4.4.1. Main Effect Test

The hierarchical regression results are shown in Table 4. The entrepreneurship education received by employees in colleges and universities has a significant positive impact on their workplace creativity (M2: *β* = 0.364, *P* < 0.001); H1 has been verified.

#### 4.4.2. Mediating Effect Test

This study draws on the regression method proposed by Baron and Kenny [27] to test the mediating effect of borderless mental model and organizational mobility preference between entrepreneurship education and creativity. The regression results are shown in Table 4. Firstly, the hypothesis that independent variable entrepreneurship education has a significant positive impact on dependent variable creativity has been supported in the main effect test. Secondly, the independent variable entrepreneurship education has a significant positive impact on the intermediary variable borderless mental model (M2: *β* = 0.440, *P* < 0.001); H2 has been verified. At the same time, the independent variable entrepreneurship education has a significant negative impact on the mediating variable organizational mobility preference (M4:*β* = -0.382, *P* < 0.001); H3 has been verified. Thirdly, after controlling the independent variable entrepreneurship education, the intermediary variable borderless mental model has a significant positive impact on the dependent variable creativity (M9: *β* = 0.478, *P* < 0.001); H4 has been verified. Similarly, the intermediary variable organizational mobility preference had a significant negative effect on the dependent variable creativity (M10: *β* = −0.192, *P* < 0.01); H5 has been verified. Finally, compared with M6, M9 (0.153 < 0.364) and M10 (0.290 < 0.364) showed a smaller effect of independent variable entrepreneurship education on dependent variable creativity. In addition, after controlling the independent variable entrepreneurship education, the regression analysis of the dependent variable creativity and the mediating variable boundary-free mental model and organizational mobility preference, respectively, found that the boundary-free mental model (M11: *β* = 0.459, *P* < 0.001) and organizational mobility preference (M11: *β* = −0.122, *P* < 0.05) still had a significant impact on creativity, and the influence of entrepreneurship education on creativity became marginal (M11: *β* = 0.115, *P* < 0.1). The above results fully demonstrate that borderless mental model and organizational mobility preference have significant mediating effects; H6 and H7 have been verified.

#### 4.4.3. Double Mediating Effect Test

This study further uses the method of Preacher and Hayes [28] to test the multiple mediating effect through the process plug-in. The results are shown in Table 5. The total indirect effect of borderless mental model and organizational mobility preference is 0.185, and the confidence interval (0.124, 0.259) does not contain 0, indicating that the two mediating variables play a significant mediating role together. Among them, the indirect effect of borderless mental model is 0.151, and the confidence interval (0.098, 0.224) does not contain 0, indicating that borderless mental model plays a significant intermediary role; H6 has been verified. The indirect effect of organizational mobility preference is 0.035, and the confidence interval (0.004, 0.074) does not contain 0, indicating that organizational mobility preference plays a significant mediating role; H7 has been verified. The comparison of the role of the two mediation paths shows that the confidence interval (0.047, 0.199) does not contain 0, indicating that there is a significant difference; that is, the mediation role of borderless mental model is significantly greater than that of organizational mobility preference.

## 5. Conclusion

Based on the human capital theory and creativity component theory, this study empirically examines the direct effect of entrepreneurship education on employees' creativity in the workplace and the dual mediating effect of boundary-free mental model and organizational mobility preference based on 266 valid sample data. The results show that entrepreneurship education received in colleges and universities can significantly promote the improvement of employees' creativity. Borderless mental model and organizational mobility preference play an intermediary role between them. The impact of entrepreneurship education on creativity is expanded from college students to employees through the bridge of borderless career attitude, which effectively verifies the lag effect of entrepreneurship education in colleges and universities and the dual intermediary effect of borderless mental model and organizational mobility preference. It further expands the research on the impact of entrepreneurship education in colleges and universities and has certain theoretical value. At the same time, the conclusions of this study have brought beneficial enlightenment to entrepreneurship education and enterprise management practice in colleges and universities.

## Figures and Tables

**Figure 1:** Theoretical research model.

**Table 1:** Basic characteristic distribution of effective samples.

Project	Category	Quantity	Percentage
Gender	Male	110	41.4
	Female	156	58.6

Age	Born in 1990–1994	142	53.4
	Born in 1995–1999	124	46.6

Highest education	Junior college and below	21	7.9
	Undergraduate	110	41.4
	Postgraduate (master's and doctorate)	135	50.8

Years of work after graduation	Less than 1 year	50	18.8
	1 year and above	65	24.4
	2 years or above	72	27.1
	3 years and above	46	17.3
	4 years and above	11	4.1
	5 years and above	22	8.3

Position	Ordinary staff	186	69.9
	Management at the grassroots level	56	21.1
	Middle and senior management	24	9.0

Enterprise scale	Less than 20 people	16	6.0
	20∼50	12	4.5
	51∼100	29	10.9
	101∼200	17	6.4
	More than 200 people	192	72.2

Nature of enterprise ownership	State-owned enterprise	67	25.2
	Private enterprise	125	47.0
	Other	74	27.8

**Table 2:** Mean value, standard deviation, and correlation analysis of main variables.

Variable	Mean value	Standard deviation	1	2	3	4	5	6	7	8	9
(1) Gender	0.411	0.493									
(2) Age	1.534	0.5	0.065								
(3) Highest education	2.429	0.636	−0.05	0.192^*∗∗*^							
(4) Working years	2.883	1.44	0.105	0.323^*∗∗*^	−0.473^*∗∗*^						
(5) Position	1.391	0.648	0.153^*∗*^	0.064	−0.298^*∗∗*^	0.478^*∗∗*^					
(6) Enterprise scale	4.342	1.2	0.002	0.128^*∗*^	0.316^*∗∗*^	−0.152^*∗*^	−0.197^*∗∗*^				
(7) Entrepreneurship education	3.203	0.821	0.095	0.036	−0.09	0.068	−0.038	−0.187^*∗∗*^			
(8) Borderless mental model	3.608	0.612	0.089	0.059	0.02	0.018	0.036	−0.094	0.442^*∗∗*^		
(9) Organizational mobility preference	2.685	0.681	−0.157^*∗*^	0.03	0.118	−0.099	−0.128^*∗*^	0.048	−0.365^*∗∗*^	−0.287^*∗∗*^	
(10) Creative ability	3.602	0.612	0.214^*∗∗*^	0.076	−0.029	0.096	0.107	−0.035	0.377^*∗∗*^	0.563^*∗∗*^	−0.316^*∗∗*^

**Table 3:** Results of confirmatory factor analysis.

Model	Factor	*χ * ^2^/Df	GFI	CFI	TLI	RMSEA
Benchmark model	Entrepreneurship education, borderless mental model,organizational mobility preference, and creativity	1.807	0.93	0.966	0.957	0.055
Competition model 1	Single factor	10.904	0.602	0.551	0.476	0.193
Competition model 2	Zero factor	19.919	0.345	0	0	0.267
Competition model 3	Merging entrepreneurship education and borderless mental model	5.121	0.775	0.82	0.782	0.125
Competition model 4	Merging entrepreneurship education and organizational mobility preferences	5.569	0.74	0.8	0.758	0.131
Competition model 5	Merging borderless mental models and organizational mobility preferences	6.45	0.719	0.761	0.712	0.143
Competition model 6	Merging borderless mental models and creativity	4.19	0.819	0.86	0.831	0.11
Competition model 7	Merging organizational mobility preferences and creativity	6.17	0.725	0.774	0.727	0.14

**Table 4:** Hierarchical regression analysis.

Variable	Borderless mental model		Organizational mobility preference		Creative ability						
	M1	M2	M3	M4	M5	M6	M7	M8	M9	M10	M11
Gender	0.079	0.032	−0.154^*∗*^	−0.113+	0.194^*∗∗*^	0.155^*∗∗*^	0.151^*∗∗*^	0.148^*∗*^	0.140^*∗∗*^	0.133^*∗*^	0.127^*∗*^
Age	0.065	0.044	0.032	0.051	0.038	0.02	0.002	0.047	−0.001	0.029	0.006
Highest education	0.03	0.039	0.072	0.064	0.044	0.051	0.027	0.065	0.032	0.063	0.041
Working years	−0.033	−0.055	−0.033	−0.013	0.034	0.015	0.052	0.024	0.042	0.013	0.039
Position	0.017	0.079	−0.071	−0.124+	0.054	0.104	0.044	0.032	0.067	0.081	0.053
Enterprise scale	−0.112+	−0.029	−0.004	−0.075	−0.025	0.043	0.035	−0.027	0.057	0.028	0.047
Nature of enterprise 1	0.042	0.051	0.079	0.071	0.03	0.038	0.007	0.054	0.014	0.052	0.023
Nature of enterprise 2	0.093	0.044	0.095	0.137^*∗*^	0.153^*∗*^	0.113	0.103+	0.181^*∗∗*^	0.092	0.139^*∗*^	0.109+
Entrepreneurship education		0.440^*∗∗∗*^		−0.382^*∗∗∗*^		0.364^*∗∗∗*^			0.15 3^*∗∗*^	0.290^*∗∗∗*^	0.115 +
Borderless mental model							0.542^*∗∗∗*^		0.478^*∗∗∗*^		0.459^*∗∗∗*^
Organizational mobility preference								−0.30^*∗∗∗*^		−0.192^*∗∗*^	−0.122^*∗*^
Fitting index											
*F*	0.935	7.443^*∗∗∗*^	1.710+	6.473^*∗∗∗*^	2.579^*∗∗*^	6.956^*∗∗∗*^	15.987^*∗∗∗*^	5.399^*∗∗∗*^	15.464^*∗∗∗*^	7.463^*∗∗∗*^	14.720^*∗∗∗*^
*R * ^2^	0.028	0.207	0.051	0.185	0.074	0.196	0.36	0.16	0.377	0.226	0.389
△*R*^2^	—	0.179	—	0.135	—	0.122	0.285	0.085	0.181	0.03	0.193

**Table 5:** Test results of double mediating effect.

Category	Effect value	Standard error	Lower 95% confidence interval	Upper 95% confidence interval
Indirect total effect	0.185	0.034	0.124	0.259
Indirect effects of borderless mental models	0.151	0.031	0.098	0.224
Indirect effects of organizational mobility	0.035	0.018	0.004	0.074
Indirect effect difference	0.116	0.038	0.047	0.199

## Data Availability

The experimental data of this research are available from the corresponding author upon request.
